# Design of the Internet plus Drug Circulation Business Model Based on Value Chain

This article has been retracted.

**DOI:** 10.1155/2021/6673649

**Published:** 2021-04-12

**Authors:** Linmeng Liang

**Affiliations:** Xijing University, Xi'an 710123, Shanxi, China

## Abstract

With the continuous development of computers and the Internet, all industries in China have brought new opportunities for change, and pharmaceutical e-commerce has also shown great potential for development. With the call and encouragement of national policies, the “Internet + drug distribution” business model has shown great potential to replace the traditional drug distribution model in the near future due to its advantages of shortening the transaction process and reducing the cost of enterprises. This paper presents a literature review on theories related to “Internet + drug distribution,” value chain and business model at home and abroad, and focuses on how traditional drug distribution enterprises should adopt the “Internet + drug distribution” model when the country is vigorously promoting it. The study focuses on how traditional pharmaceutical distribution companies should innovate their business models from the perspective of value chain to seek better development. By comparing the business models before and after the innovation, the new business model of “Internet + drug distribution” can help enterprises establish diversified value propositions, increase revenue channels, and reduce operating costs. At the same time, it can integrate and innovate the internal and external value chains of enterprises, so that traditional pharmaceutical distribution enterprises can further enhance their competitiveness and expand their market share. This thesis can enrich the application of value chain and business model theories in the field of “Internet + drug distribution,” and it is hoped that the model experience developed in this thesis can be used as a reference for similar enterprises in their transformation process.

## 1. Introduction

### 1.1. Research Background

The National Development and Reform Commission, the Ministry of Commerce, and other departments jointly issued a number of policy documents in 2019, including the “Action Plan for Promoting the High-Quality Development of the Health Industry (2019–2022),” which particularly emphasizes that the state will actively pilot the development of “Internet + drug circulation” business model. It encourages pharmaceutical distribution enterprises, medical institutions, and e-commerce enterprises to actively cooperate in the pharmaceutical distribution industry to vigorously promote cloud computing, big data, Internet of Things, and other emerging technologies, under the premise of legal compliance, simplify drug transactions and drug distribution process, and improve the efficiency of the circulation of drugs. At the same time, it encourages enterprises in a position to carry out technology development, relying on independent APP or WeChat applet and other forms of online consultation platforms, so that drug stores can support the video opening prescription. At the same time, with the help of O2O and other services, it provides convenient drug online purchase services to the majority of consumers.

According to the research data of AiMedia Data Center (as shown in Figure 1), the total B2C model sales of China's medical e-commerce industry reached 98.424 billion yuan in 2019, with a year-on-year growth rate of 61.1%, indicating that consumers have gradually developed the habit of purchasing pharmaceutical goods through online channels, and the market scale of pharmaceutical e-commerce is currently growing in a straight line; all these data fully indicate that China's traditional drug distribution model is not enough in the face of the rapid development of the Internet and needs to be transformed to the “Internet + drug distribution” model with the support of information technology.

After researching and understanding, the traditional drug distribution in China has too many communication links, including agents at all levels, logistics and distribution, and terminal sales. The increase of links means the increase of cost. These links lead to the inflated final price of drugs, and the marketing cost, R&D cost, and operation cost of drug distribution-related enterprises are also increasing, but the sales profit cannot be effectively guaranteed. Although these problems have been alleviated to a certain extent with the promotion of the “two-ticket system” policy, in this context, how to further reduce the cost and gain more profit is a key concern for many pharmaceutical companies. The “Internet + drug distribution” model can effectively help drug distribution enterprises to increase their core competitiveness, improve management efficiency and management level, and ultimately achieve the purpose of revenue diversification and cost reduction. In this paper, the feasibility of “Internet + drug distribution” business model and the specific implementation path are studied for the current situation of drug distribution model development.

### 1.2. Research Methods

In this paper, the main methods used in the research process include two kinds, namely, literature research and comparative analysis:

1. *Literature Research method*. This paper combs the literature of “Internet plus drug circulation,” value chain and business model theory, and provides theoretical support for the follow-up research on business model innovation based on value chain perspective.
2. *Comparative Analysis*. By comparing and analyzing the value chain of the Internet plus drug circulation business model before and after the construction of the pharmaceutical company, we can make a more direct analysis of the business efficiency before and after the business model innovation.

### 1.3. Purpose and Significance of the Study

In the context of the new epidemic, the country attaches great importance to the construction of the public health care system, of which the importance of pharmaceutical distribution is self-evident, as an important and indispensable part of the entire public health care system. As the country promotes the “two-ticket system” and encourages the development of “Internet + pharmaceutical circulation” industry, Chinese pharmaceutical circulation enterprises are facing huge changes and adjustments. In this context, this paper takes the value chain and business model theory as the basis and takes HY pharmaceutical distribution company as the research object to conduct a case study. In the context of “Internet+” development, we hope to summarize the current situation and problems of HY's value chain and business model development and propose valuable optimization and innovation solutions to help it carry out business model innovation.

As a new industry encouraged and advocated by the state, “Internet + drug distribution” can effectively solve the problems of drug distribution enterprises in the context of “Internet+” and “two-ticket system.” Under the background of “two-ticket system,” the challenges faced by logistics, information flow, and capital flow are conducive to helping enterprises carry out model innovation from the perspective of industry chain and value chain, which is of practical significance to help drug distribution enterprises reduce costs and increase profits. The “Internet + drug distribution” business model can also be an effective solution to the problem of expensive, difficult, and troublesome drug buying for ordinary consumers, by providing online medical treatment, electronic medical records, and other services to help consumers buy the most appropriate drugs at the nearest pharmacy and through the B2C e-commerce platform, which allows consumers to shop online.

This paper explores how drug distribution enterprises can reorganize their value chain and innovate their business model under the trend of “Internet+” and the background of the national policy of “Internet + drug distribution” and find their own innovative development path, which can help traditional drug distribution enterprises to innovate their business model from the perspective of value chain and achieve cost reduction and revenue diversification.

## 2. Literature Review

### 2.1. “Internet Plus Drug Circulation”

Traditional drug circulation refers to the intermediate link that pharmaceutical enterprises deliver drugs to consumers through logistics and transportation, storage by wholesalers, and sales. The traditional drug circulation model described in this paper mainly refers to the way to realize the process from production to consumption.  Figure 2 shows the common drug circulation model in the market. The roles involved mainly include pharmaceutical manufacturing enterprises, four-level distributors, terminal sales pharmacies, and consumers, and the sales path is progressive.

“Internet plus medicine circulation” business model is a business model of pharmaceutical circulation that pharmaceutical companies can achieve online through B2C, O2O, B2B, and other business models. The emergence of this new model greatly reduced the traditional drug circulation intermediate links and made the drug circulation intermediate links continuously reduced and the consumers' purchase of drugs reduced, and the profits of pharmaceutical companies selling drugs were also guaranteed. It is a new pattern of drug circulation with multiple gains, as shown in Figure 3, which is a typical Internet plus drug circulation model.

### 2.2. Value Chain Theory

The theory of value chain was first proposed by Michael Porter, which is mainly used to analyze the competitive advantage of enterprises. The research on value chain by scholars at home and abroad mainly includes the analysis, integration, and application of value chain. Its content mainly includes the process of purchasing, producing, and selling a series of business activities, as well as the collection of various activities related to enterprise operation. The ultimate goal is to surround the production of enterprise profits.

#### 2.2.1. Analysis of the Value Chain

In the study of Zhuo and Liu (2001), it is believed that starting from the value chain, all business activities and behaviors of enterprises can be divided into basic and auxiliary activities, and they can be further divided into more detailed and accurate activities, as for the enterprise value analysis and cost analysis, business model innovation provides great help [1]. The analysis of the value chain can also be understood as the analysis of the internal and external activities of the enterprise. In the analysis process, the internal and external activities of the enterprise will be sorted out into the corresponding value chain to fully explore the core competitive advantage of the enterprise, which can be summarized as the following two parts.

(1) *Analysis of the External Value Chain of the Enterprise*. According to Yan Jinfang (2013), as a link in the value chain, enterprises can use the external value chain to control environmental costs from the outside and pay close attention to the upstream and downstream partners in the external value chain, so that the internal and external value chains of enterprises can be effectively connected to form a closely linked whole-life process chain and finally achieve the purpose of reducing the operating costs of enterprises.

(2) *Internal Value Chain Analysis*. Liu (2011) found that the main purpose of the internal value chain analysis is to identify the enterprise's own value chain and its strengths and weaknesses and to build an internal value chain based on it. The internal value chain analysis mainly includes the following three steps: firstly, identifying the internal value chain and attributing costs; secondly, analyzing the cost drivers and decomposing the three major cost areas; finally, identifying the relationship between each link of the internal value chain and forming the enterprise cost chain system.

#### 2.2.2. Integration of the Value Chain

Su Yingshan (2020) found that, in the integration of enterprise value chain, the internal and external integration degree and matching degree of value chain are important forms of enterprise boundary change and selection. In the process of internal value chain integration, more attention is paid to the integration of enterprise core resources, while the integration of external value chain mainly improves the ability boundary of enterprises through the integration of external resources [2].

#### 2.2.3. Application of Value Chain

According to Tuling (2020) from the perspective of value chain, marketing is no longer a “certain link” of enterprise production and management, but the whole process of enterprise management. Therefore, feed enterprises should analyze the new feed marketing environment from a comprehensive perspective, actively build integrated marketing, and differentiate marketing and precise “big marketing” strategy, so as to enhance the brand influence of feed enterprises and effectively expand the market share of feed products [3].

### 2.3. Business Model Theory

#### 2.3.1. Connotation of Business Model

In 1957, foreign scholar Bellman, Clark first quoted the term business model in his paper. Slywotzky (1996) pointed out that the business model is a way for enterprises to select target customer groups, find their consumption pain points, conduct differentiated positioning with products or services, then determine marketing promotion strategies, and ultimately create value for customers and obtain theory for enterprises [4]. Rappa (2004) believes that business model is the method of company management. The company uses the relevant strategies of business model management to allocate internal and external resources, control enterprise costs, maximize customer value, and finally earn profits and benefits [5]. Zhu and Lin (2015) believe that, in the process of business model research based on value chain, it is necessary to strengthen in-depth mining, especially the problem of internal business process optimization, and the business model research for value network pays more attention to horizontal extension, aiming at expanding the contribution of enterprise value. The two complement each other, which can reveal the value logic of business model more comprehensively [6].

#### 2.3.2. Business Model Canvas

Business model as an analysis method is widely circulated in the enterprise industry, which can help enterprises to comprehensively and fully sort out each main component of the business model and sort out the circulation relationship between each link in the business model, and on the basis of the analysis results, it can become the main reference basis for enterprises to further optimize their business model and carry out business model innovation, cost control, and optimization. Combined with the main processes of business model operation, the business model canvas can be formed by arranging and combining according to the logic of business operation, which can show the advantages and disadvantages of the business model of the enterprise very intuitively. The original template of the business model canvas is shown in Figure 4.

### 2.4. S2B2C Business Model

S2B2C business model was proposed by Professor Zeng Ming of Lakeside University, which evolved from the traditional B2B model, as shown in Figure 5. This model has experienced the B2B1.0 information model and the B2B2.0 transaction model. It has developed from the transactional industry Internet. It connects major suppliers, distributors, and customers on the basis of traditional transactions. It is a brand new e-commerce marketing model that helps to improve the efficiency of commercial circulation, the product circulation supervision system, and customer service.

## 3. Analysis on the Value Chain of Traditional Medicine Circulation Enterprises

According to the research data of Aimedia Data Center (Figure 6), the total sales volume of B2C model in China's medical e-commerce industry reached 98.424 billion yuan in 2019, with a year-on-year growth rate of 61.1, indicating that consumers have gradually developed the habit of purchasing pharmaceutical products through online channels, and the market scale of pharmaceutical e-commerce is currently growing in a straight line. These data show that the business model of China's pharmaceutical retail industry is about to change, and the traditional pharmaceutical distribution model is not enough in the face of the rapid development of the Internet and needs to transform to the “Internet + pharmaceutical distribution” model with the support of information technology.

Through the comparative analysis of public data of listed companies, it is concluded that the value chain of traditional drug circulation enterprises is shown in Figure 7.

### 3.1. External Value Chain

The external value chain of drug distribution companies mainly includes suppliers, customers, complements (partners), and competitors [7]. Suppliers include drug raw material suppliers and drug suppliers (traditional Chinese medicine, Western Medicine), which are important components of the external value chain of drug distribution companies and are responsible for providing basic production materials to the company. Customers are mainly located in hospitals or retail pharmacies with end-users. The marketing activities of drug distribution companies mainly focus on this customer group. Therefore, a series of marketing promotion plans are designed, including marketing advertisements for end-users. Customer can also directly obtain relevant services through the existing B2C e-commerce system of drug distribution companies to purchase drugs.

### 3.2. Internal Value Chain

According to Porter value chain, the internal value chain of drug distribution companies includes two parts: main activities and supporting activities. The main activities include the supply of pharmaceutical raw materials, pharmaceutical production, pharmaceutical circulation and product distribution for distributors, and the key points of marketing and channel distribution. Support activities include medical human resource management, logistics distribution, and technology research and development, which lay a good foundation for the main activities [8].

## 4. Analysis on Business Model of Traditional Drug Circulation Enterprises

The existing business model of traditional drug distribution companies can be simply summarized as follows: through self-built logistics and warehousing channels, based on downstream distribution channels and self-operated stores, it provides drug circulation services, obtains sales expenses, and realizes profits [9]. By summarizing the elements of the company's business model, the business model canvas can be obtained through canvas modeling, as shown in Figure 8.

### 4.1. Necessity of Building the Internet plus Drug Circulation Business Model

Although the existing business model of traditional drug distribution enterprises has some innovation, in the face of growing customer demand, there are some problems, such as the weakening of value proposition advantage, the challenge of operation mode, the single content of customer interface, and the continuous decline of profitability. These risks are the necessity to build the innovation and transformation of the “Internet + drug circulation” business model and are also the direction to promote the business model innovation of drug circulation companies [10].

#### 4.1.1. The Advantage of Value Proposition Is Weakened

(1) *The Advantage of Value Proposition Is Gradually Weakened*. The original value proposition of traditional drug distribution enterprises focuses on the “speed” of drug distribution. In the initial stage, it realizes its dominant position by establishing logistics distribution center, warehouse distribution center, and other related means and economic investment. However, this business model has strong replicability [11]. With the continuous influx of capital, the backward enterprises can easily establish more complete, higher distribution efficiency, and better service experience through warehousing investment, team building, personnel recruitment, and other ways, so that the value proposition advantage of traditional drug circulation enterprises is gradually weakened.

(2) *Expansion of New Market Fails to Meet Expectations*. With the local market share of traditional drug distribution enterprises gradually full, it is inevitable to expand the new market in the national field, but this part of work is still unsatisfactory [12]. There are two main reasons: first of all, most of the rest of the country are the markets that competitors have been cultivating for many years, so it is too difficult for outsiders to take a share. Secondly, with the vigorous development of the Internet industry, more and more capital has been invested in Internet drug distribution companies [13]. These new companies carry out business model transformation and integrate resources by means of opening and win-win results. They can carry out business at a lower cost, causing a huge threat of competition, and even encroach on the local market share of traditional drug circulation enterprises and give to the public. They have brought great development pressure.

#### 4.1.2. Business Model Faces Challenges

Traditional drug distribution enterprises rely on the direct marketing model, which is facing the impact of the new operation mode of other drug distribution enterprises. In recent years, the continuous influx of Internet capital into the drug circulation industry has caused great challenges to the company's operation mode. For example, Haoyao business network operated by Kangning Yisheng Pharmaceutical Technology Co., Ltd., adopts the customized service of ERP + B2B, which helps commercial companies build a seamless connection between internal ERP data and pharmaceutical B2B e-commerce mall and paves the way for the transformation and upgrading of commercial companies and leapfrog development [14]. In contrast, traditional drug distribution enterprises, although they have certain business model innovation and upgrading, cannot be like the good drug business network to develop the market and business in a larger pattern [15].

#### 4.1.3. The Content of Customer Interface Is Single

At present, the content of customer interface of traditional drug distribution enterprises is relatively simple, and it is only open to distributors' customers. Distributors can simply order, receive, and query through relevant platforms. Compared with emerging drug distribution enterprises, especially Internet drug distribution enterprises, distributors are not so good [16]. Single content of customer interface means that the value provided by enterprises for customers is limited, and the added value gained by consumers in purchasing goods is relatively small. It is easy to reduce the consumption experience of users and make customers turn to other competitors.

#### 4.1.4. Profitability Continues to Decline

(1) *Risk of Revenue Decline*. With the rapid development of old competitors and the capital injection of Internet drug circulation enterprises, the original market share of traditional drug distribution enterprises is facing the risk of decline. At the same time, with the entry of competitors and the emergence of alternative drugs, the original product sales profit and customer unit price cannot be guaranteed, and the following may be the development trend of income decline. If the crisis cannot be contained effectively, it will bring greater risks to enterprises [17].

(2) *Risk of High-Cost Expenditure*. With the continuous expansion of competitive pressure, traditional drug distribution enterprises have to continue to increase capital investment in the construction of logistics distribution system, marketing promotion, and other aspects [18]. These high-cost expenditures are currently facing the problem of disproportionate expenditure and income, which is a relatively low-efficiency means of competition and is not conducive to the development of the company.

### 4.2. Innovative Internal and External Environments for Business Models of Traditional Pharmaceutical Distribution Companies

#### 4.2.1. External Environment for Business Model Innovation of Traditional Drug Distribution Enterprises

The development of information technology provides unlimited possibilities for business model innovation. The promotion of the “Internet plus” strategy has gradually satisfied people's diversified consumption needs. The most direct way is the transformation of consumption patterns and shopping methods. Consumers have developed consumption habits with the characteristics of the times under the training of all kinds of Internet applications, and the whole society has gradually recognized it [19]. It can bring about industrial change, consumption change, and mode change brought by “Internet plus” technology. Taking the field of travel as an example, there were only two types of travel modes: self-driving and public transportation [20]. Now, there are emerging business models such as bike sharing, car sharing, and online car rental. At the same time, the ways of buying tickets are gradually diversified. You can buy tickets through various channels other than official channels [21]. At the same time, online automatic ticket grabbing and self-determination time are also available to some extent; the user experience is even higher than the original software. For the pharmaceutical field, people have been able to accept the purchase of drugs through well-known and guaranteed online platforms such as Jingdong pharmacy. With the promotion of large hospitals, online consultation and video diagnosis and treatment have gradually been recognized by consumers [22].

At the same time, China has long attached great importance to the technical innovation of the medical industry. Through various policy guidance, we encourage qualified enterprises to actively carry out model innovation exploration, play a model role for similar enterprises, encourage enterprises to speed up technological innovation, and carry out business model reform and innovation with new technology and new format. Therefore, more and more pharmaceutical production enterprises and drug circulation enterprises have been established. Drug distributors will start to promote the construction of the Internet platform and try to grasp market opportunities. This is a rare opportunity and challenge for traditional drug circulation enterprises. The business model innovation of “Internet plus drug circulation” should be regarded as an important strategic plan for enterprises to meet consumers' needs for diversified drug purchase channels and actively promote innovation.

#### 4.2.2. Internal Environment of Business Model Innovation of Traditional Drug Distribution Enterprises

Traditional drug distribution enterprises have followed the development trend of the times and market reform and have actively moved closer to the Internet field. They have opened exclusive direct stores in Tmall and Jingdong. In the subsequent development, they have gradually expanded the functions of WeChat public platform and mobile phone mall, which have a certain foundation of Internet marketing.

For the online business module, some companies for the development of online business are equipped with a special business team, the necessary network marketing operations, artists, and developers. At present, the online shopping mall and WeChat platform have a primary function development and a more comprehensive product system. At the same time, in order to carry out the related business smoothly, most companies have established a free logistics distribution system locally, which can ensure the rapid, safe, and convenient distribution of related drugs to consumers and suppliers, reduce the intermediate links, and improve the operation efficiency.

To sum up, in view of the innovation of the business model of “Internet plus drug circulation,” the traditional pharmaceutical circulation enterprises have formed a good internal innovation environment, which has a good implementation basis and has internal supporting conditions for docking and merging with the “Internet plus” system.

## 5. The Path of Business Model Innovation from the Perspective of Value Chain

### 5.1. Value Proposition Innovation: Customer Diversification and Marketing Promotion

#### 5.1.1. Redefining Target Customers

Customers are the core resources in the process of enterprise market expansion. How to further clarify customer portraits, tap more customer needs, and develop a broader customer market on the basis of meeting existing customer needs is a very critical activity. Enterprises can carefully analyze and compare the existing customer base through questionnaire survey, market competition research, and other means, summarize the current situation of the existing customer base, put forward new demands, and expand the scope of target customer groups in combination with the market development law and the industry development law, so as to provide customer base guarantee for enterprises to further increase market share.

#### 5.1.2. Value Content Innovation

The products and services provided by enterprises to target customer groups must be valuable and targeted to solve the pain points of target customer groups. In the process of product and service design, enterprises should adhere to the goal orientation, take the common pain points of target customer groups as the starting point, carry out product and business innovation design, maximize customer service experience, strive to help users solve the pain points more and more comprehensively on the basis of value orientation and cost priority, and provide valuable and warm services. We should constantly promote technological innovation and innovate the value content according to the development of the times.

#### 5.1.3. Innovation of Value Transmission Mode

How to push valuable services and products to customers in need is a topic worth studying. In the vast majority of markets, there is the problem of improper value transmission, which leads to customers unable to pay for products and services. Market changes, industry development, and changes in target customers groups may bring about the demand for updating the value transfer mode. If enterprises want to transfer value to customers more quickly and accurately, they need to innovate the way of value transmission, such as the creation of marketing channels. Since 2019, the development of media has been rapid, with short video TikTok as the representative of short video platform. This has become the main way for many enterprises to carry out marketing promotion and spread value.

### 5.2. Innovation of Operation Mode: Reconstruction of Internal Business Process

From the overall point of view, the operation mode of the enterprise stipulates the process of each project business and the communication and cooperation relationship between the internal departments. Determination of the operation mode is very important for the development of enterprises. In addition to making enterprises better meet the needs of customers, it can also better play the advantages of enterprises, carry out in-depth cooperation with upstream and downstream customers, and maximize the value of the industrial chain. At the same time, the enterprise internal business process update, comprehensively sort out and upgrade the original production structure and organization and management system, which can break the gap between the original operation modes of various decentralized entities, make full use of all enterprise resources, improve the operation efficiency of enterprises, and exert enterprise value.

### 5.3. Interface Mode Innovation: Integration of External Value Chain

The operation and development of enterprises cannot be done behind closed doors. The development and growth of enterprises need the cooperation of all links in the supply chain, especially competitors and customers. Considering this problem from the external value chain of enterprises, seeking more cooperative relations with external resources of enterprises and integrating resources can maximize the enterprise value and make the business model of enterprises clearer.

#### 5.3.1. Diversified Innovation of Customer Interface

In the traditional business model, the relationship between enterprises and customers is relatively single, and there are often only simple business transactions. In the traditional market transaction interface, consumers buy services or products that can meet individual needs at the cost of money. But with the development of “Internet plus,” the demand of consumers is more diversified and dynamic. Enterprises should take improving service quality and consumer experience as the goal, make full use of information technology means, take network platform as the medium, expand interactive channels, and carry out diversified innovation of customer interface.

#### 5.3.2. Supplier Interface Integration Innovation

In the traditional model, the role of the supplier is relatively single and can only play the role of the transaction party. In the process of transaction, the supplier can provide the corresponding products according to the requirements of the buyer to meet the purchasing demand of the buyer and promote cooperation between the two parties. However, with the reform of the industry market and the demand for social development, business models of all walks of life have changed to some extent. The roles of suppliers and purchasers have also begun to show diversified development. From the original single purchase relationship, both sides gradually form multi-level deep cooperation to jointly provide services for downstream customers and improve customer service experience.

#### 5.3.3. Collaborative Innovation of Competitor Interface

In the traditional business logic, the competitors of the same industry often regard each other as enemies of life and death and inevitably seize the market by means of vicious competition such as price war, which will make it difficult to effectively guarantee the income of both competitors. Under the background of “Internet plus,” opening cooperation has become the main means of business expansion in all walks of life. After all, there is no permanent enemy in the commercial society, only the cooperative value and cooperation relationship that has not yet been excavated. “Internet plus” opening and information sharing make all kinds of cooperation possible. Conflicts are no longer the only theme of competitors. The relationship between the two sides of the competition is also moving towards diversified development.

### 5.4. Innovation of Profit Model: Platform Development

The profit model of all enterprises is nothing more than reducing costs and increasing revenue channels. Reducing costs can be carried out by improving the operation efficiency of enterprise internal management, reducing unnecessary expenses, and optimizing supply chain relations. There are many ways to increase revenue channels, but the innovation of the profit model has always been the pursuit of every enterprise: how to innovate the profit model, maximize the role of value chain, make the enterprise operate efficiently in every link of the value chain, and serve the profit of the enterprise. Platform-based development is an efficient way. Starting from the construction of an effective platform operation mode, effective positioning and division of labor for each participating role in the value chain, based on the construction of diversified cooperative relations, business model reconstruction, and profit model innovation can help enterprises maximize their value.

## 6. Design of the Internet plus Drug Circulation Business Model Based on Value Chain

Based on the value chain, the business model of “Internet plus drug circulation” can be summarized as follows: on the basis of the original distribution channels, the model relies on the Internet plus, big data technology, efficient warehousing and logistics system as its core resources, marketing in S2B2C model, and carrying out remote pharmaceutical services in the third-party platforms, forming an internal value chain and optimizing the cost structure. Large target customer range is to achieve the goal of enhancing profitability, ultimately reduce the circulation of drugs in the market outside the hospital, and provide efficient, convenient, and low-cost drug circulation services for consumers, hospitals, and pharmacies. The specific business model canvas is shown in Figure 9.

### 6.1. Value Proposition of Customer Diversification

#### 6.1.1. Expansion of Target Customers

Although the traditional drug distribution enterprises have a relatively stable customer group, they mainly face distributors and cannot directly face the end consumers. The new business model not only covers the original distributors at all levels, but also can be extended to all terminal drug consumers to expand the scope of target customers. It is also easy to form a consumer database and lay a foundation for further big data marketing.

#### 6.1.2. Innovation of Value Content

In the original business model, the value content of traditional drug circulation enterprises is relatively single. They only provide drug distribution services, and the distribution of drugs to distributors is finished. After the business model is innovated, it can directly provide drug sales, online consultation, and other services for terminal consumers based on remote pharmaceutical services and innovate and improve the value content.

### 6.2. Business Process Reengineering and Operation Mode Innovation Based on S2B2C

After the S2B2C model is added to the company's business process, its business management process, internal and external resources, partners, and other contents will change, so it is necessary to reconstruct the internal business process and management process of the company.

#### 6.2.1. Integration of Core Resources

Pharmaceutical distribution company uses drug production technology as the core resource to build a business network with channel providers as its branches and provide drug sales service to customers. It is necessary for traditional drug circulation enterprises to cooperate with technology development companies to build S2B2C technology platform. As shown in Figure 10, in this business model, a new e-commerce marketing model, which integrates suppliers to empower channel providers and jointly serve customers, is realized.

In the first step, as a large supplier (S), a drug distribution company is responsible for integrating upstream high-quality suppliers and sources, including self-produced branded drugs.

The second step is to provide commodity and technical and data support services by distributors (B) such as drug stores of drug distribution companies.

The third step is to assist the distributor (B) to complete the drug sales service to the customer (C). This part is directly oriented to the end drug consumer.

In this mode, drug distribution enterprises can integrate excellent drug suppliers and downstream drug distributors for centralized procurement on the basis of their own drug supply; on the other hand, drug circulation enterprises can also provide SaaS management tools and technical support to channel providers, so that they can better serve customers and improve user experience.

#### 6.2.2. Key Capability Improvement

Through the standardized supply chain and service support under the S2B2C model, companies can rely on the powerful management information system capability enabled by big data and further develop remote pharmaceutical service, electronic prescription, and other modules, so as to provide power support for the improvement of key capabilities in the process of business model transformation of drug distribution companies.

### 6.3. Interface Mode Innovation of External Value Chain Integration

#### 6.3.1. Supplier Interface Innovation

The value of the original supplier is to implement the purchase requirements of the drug distribution company, and the cooperation relationship is single. Through the establishment of the new business model, drug distribution companies can integrate the resources of brand suppliers with the company's new business processes and change the role of suppliers into partners, which can not only expand income channels for drug distribution companies, but also deepen the cooperation between them.

#### 6.3.2. Competitor Interface Innovation

In the traditional business model, competitors are often hostile. But in the new business model of drug distribution company, as a large S-end supplier, it can also purchase and distribute drugs from other original competitors. At the same time, the standardized remote pharmaceutical service and electronic prescription service can also be opened to competitors, realizing a certain degree of sharing and opening mechanism, and changing the original single competitive relationship between the two sides.

#### 6.3.3. Platform-Based Information Interaction Interface

Under the traditional business model, drug distribution companies have internal information management system, but the system is not perfect, cannot adapt to the reform and innovation of S2B2C model, and cannot cover the whole process of marketing activities. After business model innovation, S2B2C platform architecture is shown in Figure 11, which is divided into data layer, business layer, and interaction layer, which can effectively cover the whole business process for supervision.

Data layer: as the bottom layer of the technical framework, it plays a supporting role in the operation of the whole system. With data analysis engine as the core, it records, collects, and sorts out the consumption behaviors and habits of users and distributors, which paves the way for further improving customer service experience. At the same time, through the collection and collation of logistics data, it can effectively monitor the progress of logistics, optimize the enterprise's warehouse management system, and improve the management level and ability.

Business level: from the perspective of distributors, open platform customers, and individual customers, the process involved in the whole enterprise business operation process is standardized management, and the process supervision is strengthened by means of logistics monitoring and marketing system to improve the operation efficiency.

Interaction layer: as the interface to face customers, based on the standard operation mode of mobile Internet era and relying on offline stores, mobile app (WeChat applet), PC mall, and online consultation platform are built to expand business model and give full play to the role of customer service center to improve user experience and customer satisfaction.

### 6.4. Profit Model Innovation of Internal and External Value Chain Optimization

#### 6.4.1. Income Diversification

As a traditional drug distribution enterprise, the original revenue source of drug distribution company mainly includes the retail and wholesale business of pharmaceutical products, among which wholesale business is the most important source of income. After fully analyzing its internal and external value chain and business model canvas, and based on the business model innovation of S2B2C model, its profit model has been effectively expanded, as shown in Figure 12 for distributors, consumers, and open platform partners.

#### 6.4.2. Substantial Cost Savings

(1) *Saving Operating Costs*. In the original business model, the cost of drug distribution enterprises in the process of operation and management is relatively high, especially when the major e-commerce platforms have launched online drug sales services, the competition pressure of enterprises has increased sharply, and the customer acquisition cost and operation cost industry have gradually increased. The operating cost of the drug distribution company will be greatly reduced. It can change from the passive acquisition of customers to the active acquisition of courses, which saves the operating cost of the enterprise and increases the profitability and competitiveness of the enterprise.

(2) *Saving Logistics Transportation Cost*. At present, the cost of drug circulation logistics is high, the logistics capacity is tense or wasteful with market fluctuation, and the degree of specialization is low. From the perspective of drug distributors, there is an urgent need for stable logistics arrival time and appropriate prices. With the implementation of new business models, drug distribution companies can use big data forecasts to combine third-party logistics companies to reduce logistics and transportation costs.

## 7. Summary

This paper investigates and understands the current traditional drug circulation model in China and finds that there are pain points in the circulation link, cost control, and value chain carding, which need to be solved. With the development of “Internet plus” technology, it provides a new possibility for solving these problems. Then, through the literature review of business model, value chain, and other scholars' research theory, this paper summarizes the path of business model innovation from the perspective of value chain, which provides theoretical support and research basis for future research and innovation.

Through the analysis of its value chain and business model, we can understand the problems existing in the development of its traditional drug distribution company. Through the business model canvas, the value proposition, operation mode, interface mode, and profit model are summarized and analyzed. From the perspective of internal value and external value, the paper builds S2B2C business model for drug distribution company and optimizes the existing business process.

## Figures and Tables

**Figure 1:** Total sales of B2C model in China's medical e-commerce industry, 2016–2021 (unit: billion yuan).

**Figure 2:** Common drug circulation patterns.

**Figure 3:** Typical Internet plus drug circulation model.

**Figure 4:** Business model canvas.

**Figure 5:** S2B2C business model evolutions.

**Figure 6:** Total sales of B2C model in China's medical e-commerce industry from 2016 to 2021 (100 million Yuan).

**Figure 7:** Porter value chain of traditional medicine circulation company.

**Figure 8:** Business model canvas of traditional drug distribution enterprises.

**Figure 9:** “Internet plus drug circulation” business model based on value chain.

**Figure 10:** S2B2C business model of drug distribution company.

**Figure 11:** Technical framework of S2B2C basic platform of drug distribution company.

**Figure 12:** Diversified income content of new business model of drug distribution company.

## Data Availability

No data were used to support this study.
